# Impact of kidney size on mortality in diabetic patients receiving peritoneal dialysis

**DOI:** 10.1038/s41598-021-87684-z

**Published:** 2021-04-15

**Authors:** Chun-Hao Chen, Chao-Yu Chen, Mei-Ching Yu, Jen-Fen Fu, Yi-Chou Hou, I.-Kuan Wang, Yu-Hsin Chih, Cheng-Hao Weng, Wen-Hung Huang, Ching-Wei Hsu, Frederick W. K. Tam, Tzung-Hai Yen

**Affiliations:** 1 Department of Orthopedic Surgery, Chang Gung Memorial Hospital, Chiayi, Taiwan; 2 Department of Nephrology, Clinical Poison Center, Kidney Research Center, Center for Tissue Engineering, Chang Gung Memorial Hospital, Chang Gung University, 199 Tung Hwa North Road, Linkou, Taoyuan, Taipei, 105 Taiwan; 3 Division of Pediatric Nephrology, Department of Pediatrics, Chang Gung Memorial Hospital, Chang Gung University, Linkou, Taoyuan, Taiwan; 4 Department of Medical Research, Chang Gung Memorial Hospital, Linkou, and Graduate Institute of Clinical Medical Sciences, Chang Gung University, Taoyuan, Taiwan; 5 Division of Nephrology, Department of Internal Medicine, Cardinal Tien Hospital, School of Medicine, Fu-Jen Catholic University, New Taipei City, Taiwan; 6 Department of Nephrology, China Medical University Hospital, China Medical University, Taichung, Taiwan; 7 Centre for Inflammatory Disease, Department of Immunology and Inflammation, Imperial College London, London, UK

**Keywords:** Endocrinology, Nephrology

## Abstract

Although patients with diabetes mellitus mostly present with enlarged or normal-sized kidneys throughout their life, a small proportion of patients have small kidneys. This longitudinal study enrolled 83 diabetic patients treated with peritoneal dialysis (PD) between 2015 and 2019. Patients were stratified into two groups, those with enlarged or normal (n = 67) or small (n = 16) kidneys, based on their kidney sizes before dialysis. Patients with small kidney size were not only older (76.63 ± 10.63 vs. 68.03 ± 11.26 years, *P* = 0.007), suffered longer duration of diabetes mellitus (272.09 ± 305.09 vs. 151.44 ± 85.31 month, *P* = 0.006) and predominantly female (75.0 vs. 41.8%, *P* = 0.017), but also had lower serum levels of creatinine (9.63 ± 2.82 vs. 11.74 ± 3.32 mg/dL, *P* = 0.022) and albumin (3.23 ± 0.67 vs. 3.60 ± 0.47 g/dL, *P* = 0.010) than patients with enlarged or normal kidney size. At the end of analysis, 14 (16.9%) patients died. Patients with small kidney size demonstrated higher all-cause (50.0 vs. 9.0%, *P* < 0.001) and infection-related (43.8 vs. 7.5%, *P* < 0.001) mortality than patients with enlarged or normal kidney size. In a multivariate-logistic-regression model, small kidney size was a powerful predictor of mortality (odds ratio 6.452, 95% confidence interval 1.220–34.482, *P* = 0.028). Diabetic patients with small kidney size at the beginning of PD carry a substantial risk for mortality.

## Introduction

It is not uncommon to find enlarged kidneys in patients with diabetes mellitus, and the kidneys could remain large even in the advanced stage of the disease. In a Sardinian population cohort study, Piras et al.^1^ presented their data that younger age, female sex, diabetes mellitus, obesity, tall height, high waist-to-hip ratio and lower serum creatinine were significant predictors of larger kidney size. The presence of diabetes mellitus was associated with a 1.723-fold risk of having a large kidney. Moreover, Rigalleau et al.^2^ reported that large kidneys predicted poor kidney outcome in patients with diabetes and chronic kidney disease. In the second manifestations of arterial disease (SMART) study^3^, large kidney length was found to be associated with higher risk of cardiovascular events and mortality in high-risk patients, irrespective of estimated glomerular filtration rate.

Nevertheless, small kidneys could be observed in a small number of diabetic patients with chronic kidney disease. Majdan et al.^4^ reported that most of their type 2 diabetes mellitus patients with chronic kidney disease had small kidneys. Notably, Habib^5^ proposed that both kidney hypertrophy and atrophy can occur in diabetes mellitus. The early changes in diabetic kidneys are mainly due to tubular basement membrane thickening, which leads to kidney hypertrophy. On the other hand, various tubulointerstitial diseases can induce apoptosis in proximal tubular cells, causing tubular atrophy and fibrosis and ultimately kidney atrophy^5^. Furthermore, atherosclerosis and related ischemic diseases can decrease the blood supply to the kidneys, resulting in kidney atrophy^5^.

Chronic kidney disease is endemic in Taiwan; indeed, the incidence and prevalence of end-stage kidney disease (ESKD) are higher in Taiwan than in any other country^6^. In 2016, Taiwan, the United States, and the Jalisco region of Mexico reported the highest incidences of treated ESKD, with rates of 493, 378, and 355 patients per million general population, respectively. Notably, diabetes is the primary cause of ESKD in 46% of incident dialysis patients in Taiwan. Nevertheless, the majority of uremic patients in Taiwan are treated with hemodialysis rather than peritoneal dialysis (PD)^7^.

The rationale for this study was based on an important, but as yet unanswered, question that arose for many diabetic patients treated with PD in our hospital. The majority of diabetic patients had enlarged or normal kidneys when entering dialysis, whereas few diabetic patients were found to have small kidneys at the time of uremia. Therefore, this raises the question of what the impact of kidney size before dialysis on the outcomes of these patients is. Perhaps one of the potential clinical applications of small kidneys is to remind clinicians about diabetic patient care. For example, if small kidney size at the beginning of PD is found to be associated with a greater risk for infection-cause mortality, physicians should be alert of the possibility of occurrence of infection and consider early initiation of antimicrobial therapy in case of infectious symptoms and signs.

Diabetes mellitus is the most important cause of ESKD worldwide, but no work has been performed to compare outcomes of diabetic patients with enlarged or normal versus small kidney size, which initiated our interest in this research. Therefore, this study attempted to survey kidney size in diabetic PD patients before the commencement of dialysis and to analyze the association of kidney size with outcomes and laboratory biomarkers.

## Results

This study included 83 diabetic patients receiving long-term PD at Chang Gung Memorial Hospital (Table 1). Most of the diabetic patients had enlarged or normal kidney size (n = 67, 80.7%) at the beginning of PD, but some patients had small kidney size (n = 16, 19.3%) when entering PD. The patients were aged 69.70 ± 11.57. These patients had been receiving PD for 42.82 ± 3.72 months. None of the patients were on immunosuppressive medications. Many patients suffered from hypertension (90.4%) and cardiovascular disease (41.0%). It was found that patients with small kidney size were not only older (76.63 ± 10.63 vs. 68.03 ± 11.26 years, *P* = 0.007) and suffered longer duration of diabetes mellitus (272.09 ± 305.09 vs. 151.44 ± 85.31 month, *P* = 0.006), but also more often female (75.0 vs. 41.8%, *P* = 0.017) than patients with enlarged or normal kidney size.

**Table 1:** Baseline characteristics of peritoneal dialysis patients stratified by kidney size (n = 83).

Variable	All patients (n = 83)	Diabetic patients with enlarged or normal kidney size (n = 67)	Diabetic patients with small kidney size (n = 16)	*P* value
*Demographics*				
Age, years	69.70 ± 11.57	68.03 ± 11.26	76.63 ± 10.63	0.007**
Female sex, n (%)	40 (48.2)	28 (41.8)	12 (75.0)	0.017*
Biopsy-proved glomerulonephritis, n (%)	1 (1.2)	1 (1.5)	0 (0.0)	1.000
Polycystic kidney disease, n (%)	0 (0.0)	0 (0.0)	0 (0.0)	1.000
Hypertension, n (%)	75 (90.4)	61 (91.0)	14 (87.5)	0.666
Cardiovascular disease, n (%)	34 (41.0)	26 (38.8)	8 (50.0)	0.413
Chronic liver disease, n (%)	5 (6.0)	3 (4.5)	2 (12.5)	0.226
Hepatitis B virus carrier, n (%)	10 (12)	9 (13.4)	1 (6.3)	0.428
Hepatitis C virus carrier, n (%)	6 (7.2)	5 (7.5)	1 (6.3)	0.866
Body mass index, kg/m^2^	25.47 ± 3.71	25.77 ± 3.59	24.29 ± 4.09	0.154
Smoking habit, n (%)	15 (18.1)	13 (19.4)	2 (12.5)	0.519
Alcohol consumption, n (%)	7 (8.4)	6 (9.0)	1 (6.3)	0.726
Immunosuppressive medications	0 (0)	0 (0)	0 (0)	1.000
Duration of peritoneal dialysis, month	42.82 ± 3.72	39.16 ± 32.22	59.14 ± 35.33	0.701
Duration of diabetes mellitus, month	174.69 ± 1158.67	151.44 ± 85.31	272.09 ± 305.09	0.006**
*Hypoglycemic therapy*				0.455
Oral hypoglycemic agents, n (%)	59 (71.1)	47 (70.1)	12 (75.0)	
Insulin, n (%)	18 (21.7)	16 (23.9)	2 (12.5)	
Oral hypoglycemic agents and insulin, n (%)	6 (0.72)	4 (0.60)	2 (12.5)	

*P < 0.05; **P < 0.01.

Compared with patients with enlarged or normal kidney size (Table 2), patients with small kidney size had lower serum levels of creatinine (9.63 ± 2.82 vs. 11.74 ± 3.32 mg/dL, *P* = 0.022) and albumin (3.23 ± 0.67 vs. 3.60 ± 0.47 g/dL, *P* = 0.010).

**Table 2:** Laboratory findings of peritoneal dialysis patients stratified by kidney size (n = 83).

Variable	All patients (n = 83)	Diabetes patients with enlarged or normal kidney size (n = 67)	Diabetes patients with small kidney size (n = 16)	*P* value
Blood urea nitrogen, mg/dL	70.66 ± 21.58	72.25 ± 21.64	63.65 ± 19.33	0.149
Creatinine, mg/dL	11.32 ± 3.35	11.74 ± 3.32	9.63 ± 2.82	0.022*
Uric acid, mg/dL	6.73 ± 1.87	6.93 ± 1.94	5.93 ± 1.24	0.052
Sodium, mEq/L	135.11 ± 3.44	135.10 ± 3.46	135.13 ± 3.30	0.983
Potassium, mEq/L	4.12 ± 1.35	4.25 ± 1.43	3.58 ± 0.66	0.071
Corrected calcium, mg/dL	9.75 ± 0.83	9.69 ± 0.85	10.01 ± 0.70	0.162
Inorganic phosphorus, mg/dL	5.52 ± 1.63	5.70 ± 1.68	4.81 ± 1.31	0.050
Fasting glucose, mg/dL	163.06 ± 71.87	164.03 ± 75.18	156.88 ± 53.52	0.721
Glycated hemoglobin, %	7.20 ± 1.47	7.19 ± 1.48	7.23 ± 1.35	0.939
Albumin, g/dL	3.5 ± 0.53	3.60 ± 0.47	3.23 ± 0.67	0.010*
Total cholesterol, mg/dL	180.41 ± 54.90	183.45 ± 56.45	166.69 ± 44.32	0.272
Triglyceride, mg/dL	231.45 ± 257.20	231.31 ± 276.30	220.81 ± 132.98	0.883
Aspartate aminotransferase, U/L	27.65 ± 15.18	26.94 ± 14.03	30.38 ± 19.23	0.417
Alanine aminotransferase, U/L	25.23 ± 20.45	25.04 ± 21.46	27.00 ± 14.54	0.731
Intact parathyroid hormone, pg/mL	283.77 ± 239.04	287.71 ± 237.40	250.16 ± 238.26	0.572
Iron, ug/dL	66.54 ± 27.88	67.87 ± 29.31	61.50 ± 22.09	0.418
Total iron binding capacity, ug/dL	267.41 ± 62.95	272.81 ± 63.20	247.31 ± 58.54	0.146
Ferritin, ng/mL	538.06 ± 601.00	528.38 ± 637.81	554.53 ± 384.32	0.876
White blood cell count, 1000/µL	8.22 ± 2.32	8.07 ± 1.92	8.92 ± 3.54	0.188
Red blood cell count, million/dL	3.90 ± 3.76	4.02 ± 4.13	3.38 ± 0.48	0.453
Hemoglobin, g/dL	9.97 ± 1.40	10.07 ± 1.46	9.53 ± 1.27	0.179
Hematocrit, %	30.15 ± 4.18	30.43 ± 4.38	28.79 ± 3.87	0.172
Mean corpuscular volume, %	87.20 ± 6.18	86.89 ± 7.21	88.48 ± 6.83	0.427
Mean corpuscular hemoglobin, pg/cell	28.90 ± 2.51	28.75 ± 2.69	29.51 ± 2.42	0.303
Mean corpuscular hemoglobin concentration, g Hb/dL	22.15 ± 1.14	33.10 ± 1.17	33.36 ± 1.08	0.408
Red blood cell distribution width, %	15.29 ± 2.08	15.20 ± 1.91	15.83 ± 2.99	0.298
Platelet count, 1000/µL	233.87 ± 90.32	238.43 ± 89.70	212.75 ± 91.55	0.308
High-sensitivity C-reactive protein, mg/L	20.22 ± 18.05	20.93 ± 44.85	16.48 ± 19.21	0.649
Log (high sensitivity C-reactive protein), mg/L	0.83 ± 0.58	0.80 ± 0.6	0.97 ± 0.51	0.301

The data represented the last laboratory values prior to the patients being started on PD. *P < 0.05.

Table 3 shows that there were no significant differences between the groups in terms of peritoneal transporter characteristics, dialysis adequacy, residual kidney function or cardiothoracic ratio.

**Table 3:** Dialysis-related data of peritoneal dialysis patients stratified by kidney size (n = 83).

Variable	All patients (n = 83)	Diabetic patients with enlarged or normal kidney size (n = 67)	Diabetic patients with small kidney size (n = 16)	P value
Erythropoietin dose, unit/month	17,108.43 ± 6248.93	16,716.42 ± 6630.52	18,750.00 ± 4057.91	0.245
Dialysate/plasma creatinine	0.69 ± 0.11	0.69 ± 0.013	0.68 ± 0.029	0.822
*Peritoneal equilibration test*				0.517
High, n (%)	12 (14.5)	10 (14.9)	2 (12.5)	
High average, n (%)	46 (55.4)	38 (56.7)	8 (50.0)	
Low average, n (%)	21 (25.3)	15 (22.4)	6 (37.5)	
Low, n (%)	4 (4.8)	4 (6.0)	0 (0.0)	
Weekly Kt/V_urea_	2.01 ± 0.04	2.00 ± 0.39	2.06 ± 0.39	0.896
Weekly creatinine clearance rate, L/1.73 m^2^	59.52 ± 15.53	60.67 ± 16.48	54.71 ± 9.67	0.170
Normalized protein nitrogen appearance, g/kg/day	1.03 ± 0.03	1.04 ± 0.03	0.99 ± 0.06	0.426
Residual kidney function, mL/min	10.66 ± 15.41	11.98 ± 16.56	5.15 ± 7.26	0.112
Cardiothoracic ratio	0.51 ± 0.06	0.51 ± 0.06	0.51 ± 0.05	0.854

Residual kidney function was determined by urinary creatinine clearance using a 24-h urine collection method. Cardiothoracic ratio was measured by dividing the biggest transverse diameter of the heart silhouette by the length between the internal margins of the ribs at the level of right hemidiaphragm.

At the end of analysis, 14 (16.9%) patients died (Table 4). Patients with small kidney size demonstrated a higher mortality rate than patients with enlarged or normal kidney size (50.0 vs. 9.0%, *P* < 0.001). Moreover, there was more infection-related mortality in the patients with small than in those with enlarged or normal kidney size (43.8 vs. 7.5%, *P* < 0.001). The sources of infection-related mortalities were three PD-related peritonitis, three nosocomial pneumonia, two pressure sore infection, one fulminant clostridium difficile colitis, one cellulitis, one diabetic foot wound infection and one pulmonary tuberculosis.

**Table 4:** Outcomes of peritoneal dialysis patients stratified by kidney size (n = 83).

Variable	All patients (n = 83)	Diabetic patients with enlarged or normal kidney size (n = 67)	Diabetic patients with small kidney size (n = 16)	*P* value
Follow-up duration, month	28.98 ± 13.22	29.76 ± 12.69	25.69 ± 15.25	0.271
All-cause mortality, n (%)	14 (16.9)	6 (9.0)	8 (50.0)	< 0.001***
Infection-related mortality, n (%)	12 (14.5)	5 (7.5)	7 (43.8)	< 0.001***
Cardiovascular-cause mortality, n (%)	2 (2.4)	1 (1.5)	1 (6.3)	0.265
Technical failure, n (%)	30 (36.1)	24 (35.8)	6 (37.5)	0.900
Peritonitis, episode/100 months	0.90 ± 2.06	0.82 ± 2.23	1.07 ± 1.12	0.706

***P < 0.001.

In a multivariate logistic regression model (Table 5), it was revealed that small kidney size was a significant risk factor associated with mortality (odds ratio 6.452, 95% confidence interval 1.220–34.482, *P* = 0.028).

**Table 5:** Analysis of mortality using a multivariate logistic regression model (n = 83).

Variable	Univariate analysis	*P* value	Multivariate analysis	*P* value
	Odds ratio (95% confidence interval)		Odds ratio (95% confidence interval)	
Age (per 1-year increase)	1.072 (1.013–1.136)	0.017*	1.029 (0.949–1.115)	0.489
Alanine aminotransferase (per 1 U/L increase)	1.009 (0.986–1.033)	0.442		
Albumin (per 1 g/dL increase)	0.132 (0.038–0.463)	0.002**	0.589 (0.090–3.861)	0.581
Alcohol consumption (yes)	1.238 (0.137–11.169)	0.849		
Aspartate aminotransferase (per 1 U/L increase)	1.041 (1.006–1.077)	0.021*	1.018 (0.964–1.076)	0.520
Blood urea nitrogen (per 1 mg/dL increase)	0.995 (0.968–1.022)	0.696		
Body mass index (per 1 kg/m^2^ increase)	1.018 (0.871–1.190)	0.821		
Calcium (per 1 mg/dL increase)	0.782 (0.429–1.423)	0.421		
Cardiovascular disease (no)	0.316 (0.095–1.046)	0.059		
Chronic liver disease (no)	0.273 (0.041–1.809)	0.178		
Corrected calcium (per 1 mg/dL increase)	1.401 (0.685–2.867)	0.356		
Creatinine (per 1 mg/dL increase)	0.689 (0.541–0.877)	0.003**	0.780 (0.556–1.095)	0.151
Duration of peritoneal dialysis (per 1-month increase)	1.004 (0.987–1.021)	0.674		
Fasting glucose (per 1 mg/dL increase)	1.006 (0.999–1.013)	0.118		
Female sex (yes)	0.308 (0.088–1.078)	0.065		
Ferritin (per 1 ng/mL increase)	1.001 (1.000–1.001)	0.197		
Glycated hemoglobin (per 1% increase)	1.295 (0.887–1.890)	0.181		
Hemoglobin (per 1 g/dL increase)	0.593 (0.373–0.944)	0.028*	0.701 (0.387–1.270)	0.701
Hepatitis B virus carrier (no)	0.414 (0.093–1.849)	0.248		
Hepatitis C virus carrier (no)	0.369 (0.061–2.246)	0.279		
High-density lipoprotein (per 1 mg/dL increase)	0.985 (0.937–1.036)	0.555		
Hypertension (yes)	3.491 (0.728–16.743)	0.118		
High-sensitivity C-reactive protein (per 1 mg/L increase)	1.013 (0.985–1.043)	0.364		
Inorganic phosphorus (per 1 mg/dL increase)	0.776 (0.534–1.127)	0.182		
Intact parathyroid hormone (per 1 pg/mL decrease)	0.998 (0.995–1.001)	0.212		
Iron (per 1 µg/dL increase)	0.995 (0.974–1.017)	0.667		
Mean corpuscular hemoglobin (per 1 pg/cell increase)	1.180 (0.919–1.516)	0.195		
Mean corpuscular hemoglobin concentration (per 1 g Hb/dL increase)	1.394 (0.822–2.366)	0.218		
Mean corpuscular volume (per 1% increase)	1.040 (0.953–1.134)	0.384		
Peritonitis (per 1 episode/100 months increase)	1.401 (0.961–2.042)	0.080		
Platelet count (each increase of 11,000/µL)	0.989 (0.981–0.997)	0.006**	0.990 (0.980–1.001)	0.064
Red blood cell count (per 1 million/dL increase)	0.330 (0.103–1.061)	0.063		
Small kidney size (yes)	10.204 (2.801–37.037)	< 0.001***	6.452 (1.220–34.482)	0.028*
Smoking habit (yes)	3.309 (0.398–27.483)	0.268		
Sodium (per 1 mEq/L increase)	0.886 (0.741–1.060)	0.185		
Total cholesterol (per 1 mg/dL increase)	0.997 (0.986–1.008)	0.556		
Total iron binding capacity (per 1 µg/dL increase)	0.995 (0.985–1.005)	0.347		
Triglyceride (per 1 mg/dL increase)	1.001 (0.999–1.003)	0.441		
Uric acid (per 1 mg/dL increase)	1.005 (0.737–1.369)	0.977		
White blood cell (per 11,000/µL increase)	1.276 (0.993–1.638)	0.056		

*P < 0.05; **P < 0.01; *P < 0.001.

Kaplan–Meier analysis revealed that patients with small kidney size had lower cumulative survival than did patients with enlarged or normal kidney size (Fig. 1, log-rank test, chi-squared = 15.614, *P* < 0.001).

**Figure 1:** Kaplan–Meier analysis. Patients with small kidney size at the initiation of dialysis (solid line) had lower cumulative survival than patients with enlarged or normal kidney size (dashed line) (log-rank test, chi-squared = 15.614, *P* < 0.001).

## Discussion

The analytical data from this study suggested that small kidney size at the commencement of dialysis could be a risk factor for mortality in the diabetic PD population. This finding adds new knowledge to the existing dialysis literature. There was no clear explanation for the observation. Nevertheless, patients with small kidney size were not only older (*P* = 0.007), suffered longer duration of diabetes mellitus (*P* = 0.006), but also had lower serum levels of creatinine (*P* = 0.022) and albumin (*P* = 0.010) than patients with enlarged or normal kidney size. The abovementioned variables, for example older age, longer duration of diabetes mellitus, as well as malnutrition (lower blood creatinine and albumin level) could attribute to increased mortality.

Many traditional risk factors for mortality have been described in diabetes patients receiving PD. In a 2-year nationwide cohort study, Abe et al.^8^ found that glycated albumin ≥ 20.0% was associated with a decrease in survival in diabetic patients on PD. In a study of 118 diabetic PD patients, Coronel et al.^9^ disclosed that age and cardiovascular comorbidity are the factors associated with mortality. In a retrospective study, Chung et al.^10^ revealed that old age, female sex, the presence of cardiovascular disease or protein-energy wasting and low residual kidney function were predictors of mortality in diabetic PD patients. In a study of 2798 diabetic PD patients, Duong et al.^11^ reported that poor glycemic control was associated incrementally with higher mortality. In a study of 61 diabetic PD patients, Koc et al.^12^ showed that hypoparathyroidemia, hypocalcemia and hypoalbuminemia were risk factors associated with mortality. In a 5-year cohort study of 809 diabetic PD patients, Yang et al.^13^ reported that older age and the presence of cardiovascular disease, hyperglycemia, anemia and hypoalbuminemia were important risk factors for mortality. In another study of 200 diabetic PD patients, Peng et al.^14^ showed that increased glycated hemoglobin and decreased albumin-corrected glycated serum protein were associated with mortality in diabetic PD patients.

Patients with small kidney size were older than patients with enlarged or normal kidney size (*P* = 0.007). Many groups have confirmed such a positive association between decreasing kidney size and aging^15–18^. Hommos et al.^16^ reported that aging could be associated with considerable changes in kidney parenchymal structure, even in the absence of age-related comorbidities. Gross pathology examination of aged kidneys found a decrease in kidney cortical volume, an increase in surface roughness, and an increase in the number and size of simple kidney cysts with aging. Histopathology examination also found an increase in nephrosclerosis (arteriosclerosis/arteriolosclerosis, global glomerulosclerosis, interstitial fibrosis, and tubular atrophy) associated with the aging process.

Patients with small kidney size were more often female than patients with enlarged or normal kidney size (*P* = 0.017). This positive association between small kidney size and female sex has been confirmed by many independent studies^17,18^. In a study of 665 adult volunteers, Emamina et al.^17^ reported a sex difference in kidney size in adults; the median kidney lengths were 11.0 cm (women) and 11.5 (men) on the left side and 10.7 cm (women) and 11.2 cm (men) on the right side. Therefore, the female kidney was usually smaller than the male kidney. On the other hand, Piras et al.^1^ revealed that female sex was associated with a 2.035-fold risk of having a large kidney. Finally, it was unclear whether the diabetic females had more history of analgesic use than diabetic males, although there were no medical records for this, and the recall history was subjected to memory bias. A questionnaire survey in Norway revealed^19^ that women used both more nonprescription analgesics and more prescription analgesics than men.

The average age of patients in this study was 69.70 ± 11.57 years. This figure is close to that of the Japanese study. In Japan, patients are approximately 69 years of age at the initiation of dialysis^20^. Currently, there has been a trend of shifting from hospital-based care of older patients to home-based care. Assisted PD has been promoted as an alternative method for older patients with ESKD^21^. Older patients are susceptible to many physiological changes related to aging and problems such as anxiety, depression, dementia, visual impairment, and cognitive impairment, all of which impede self-performance of PD. Assistance from home-care nurses or assistance from a younger family member may be the solution. In a study of 128 Japanese PD patients, Sakai and Nihei^20^ reported that the older group (≥ 70 years of age) did not show higher rates of technical failure, but their survival was shorter than that of the younger group (< 70 years of age). In Taiwan, most families are large families, with three generations living in the same household. Younger family members can take care of their older parents and assist them in performing PD therapy. This may explain the higher age of PD in this study.

Patients with small kidney size patients suffered from lower serum levels of creatinine (*P* = 0.022) and albumin (*P* = 0.010) than patients with enlarged or normal kidney size. Albumin is the most abundant protein in human serum^22^. Albumin is produced by the liver and is an indicator of malnutrition. On the other hand, creatinine is the end product of creatine, is mainly present in skeletal muscle and is used as a surrogate measurement of muscle mass^23^. Creatinine generation is reduced in the setting of low skeletal muscle mass, such as in older patients. Since patients with small kidney size were older and with a predominance of females, it was not surprising that these patients had lower serum levels of creatinine and albumin than the enlarged or normal kidney size group.

Patients with small kidney size demonstrated higher all-cause (*P* < 0.001) and infection-related (*P* < 0.001) mortality than patients with enlarged or normal kidney size. Diabetics generally have an increased propensity to develop infections. The increased occurrence of infections in diabetic patients is caused by the hyperglycemic milieu, which supports immune dysfunction (such as the impairment of neutrophil function, the suppression of antioxidant system, and humoral immunity), angiopathy, neuropathy, a decrease in the antibacterial activity of urine, gastrointestinal and urinary dysmotility, and an increased need for medical interventions^24^. Diabetes impairs antibacterial defenses and increases the risk of infection^25^. Furthermore, a high concentration of glucose degradation products in PD solutions could accelerate leucocyte apoptosis and damage peritoneal antibacterial defense^26^. Previous studies^27,28^ have reported diabetes mellitus as a risk factor for PD-associated peritonitis. According to a large retrospective cohort study in China^29^, peritonitis was always associated with a higher risk of mortality in PD patients, and its influence on mortality was more significant in patients with longer PD durations. The assessment of the immune defense system of the diabetic patients with small kidney size will need further investigation.

The limitations of this study included small sample size and short follow up duration. In addition, the relationship between small kidneys and mortality was simply a correlation, rather than causal relationship. Since this study involves retrospective review of existing data, it is impossible to make a causal relationship conclusion. The pathophysiological mechanism by which small kidneys confer increased infection risk cannot be answered by this study. Although patients with small kidney size were older and suffered longer duration of diabetes mellitus than patients with enlarged or normal kidney size, there were no difference in blood sugar control between both groups, which could confer increased infection risk. This study is also limited by lacking protocol kidney biopsy. Since approximately half of cases of ESKD in Taiwan are due to diabetic nephropathy, it is possible that half of this cohort may have had other kidney diseases. All patients in this study are diabetes, but the etiologies of renal failure are varied. Since kidney biopsy remains an invasive procedure, it is usually not considered a routine in patients with diabetes mellitus unless suspicion of non-diabetic renal disease. As shown in Table 1, only one patient received kidney biopsy and the pathology report revealed co-existing glomerulonephritis. Further prospective studies are warranted to confirm this finding.

## Conclusion

In summary, small kidney size at the beginning of dialysis carries a substantial risk for mortality in diabetic PD patients. These patients demonstrated higher all-cause and infection-related mortality than patients with enlarged or normal kidney size.

## Methods

### Inclusion and exclusion criteria

All diabetic patients aged 18 years and above receiving chronic PD at Chang Gung Memorial Hospital between 2015 and 2019 were included in this study. Patients who had been receiving PD for less than 6 months; those who had been hospitalized or operated on or who had received a kidney transplant in the preceding 3 months; and those with cancer were excluded from the study (Fig. 2).

**Figure 2:** Flow chart. Diagram shows the enrolment and status of patients. *ESKD* end-stage kidney disease, *PD* peritoneal dialysis.

### Groups

Patients who met the inclusion criteria were divided into two groups according to their kidney size when entering PD. All patients received ultrasonographic evaluation of kidney size and echogenicity, and a small kidney was defined as when the kidney length was less than 9.0 cm^4^.

### PD prescription

PD prescriptions were based on the peritoneal membrane characteristics determined by the peritoneal equilibration test^30^. Intermittent therapy was prescribed to patients with high membrane transport and continuous therapy and to those with average or low membrane transport. Low-calcium (1.5 or 1.25 mmol/L), icodextrin-based (7.5 g/dL) or standard dialysates containing glucose (sodium, 135 mmol/L; lactate, 35 mmol/L; calcium, 1.75 mmol/L) were used according to the patients' peritoneal transport characteristics and serum calcium levels to maintain adequate ultrafiltration and enlarged or normal calcium levels. Dialysis prescription aimed at obtaining a total Kt/V of at least 1.8 per week.

### Laboratory analysis

The data represented the last laboratory values prior to the patients being started on PD. All laboratory values, including blood cell count, biochemical data, dialysate/plasma creatinine ratio, peritoneal transport characteristics, weekly creatinine clearance and weekly Kt/V_urea,_ were surveyed by automated and standardized methods. All blood samples were collected in the morning after at least 10 h of fasting. Serum levels of calcium, phosphate and intact parathyroid hormone were also surveyed, and the corrected serum calcium level was calculated as calcium (mg/dL) = [0.8 (4.0 − albumin[g/dL])]. All other markers were surveyed via standard laboratory methods using an automatic analyzer.

### Statistical analysis

The continuous variables are presented as the means ± the standard deviations for the numbers of observations, whereas the categorical variables are presented as numbers (percentages)^31^. For comparison between two groups, Student's t-test was used for quantitative variables, whereas the chi-squared or Fisher's exact test was used for categorical variables. Survival data were analyzed with the Kaplan–Meier method and tested for significance using the log-rank test. A univariate binary logistic regression analysis was performed to compare the frequency of potential risk factors associated with mortality. To control for confounders, a stepwise backward multivariate binary logistic regression analysis was performed to analyze the variables that were significant on univariate analysis. The criterion for significance to reject the null hypothesis was a 95% confidence interval. The statistical analyses were performed using IBM SPSS Statistics Version 25 for Mac (IBM corporation, Armonk, NY, USA).

### Ethical statement

This longitudinal observational study complied with the guidelines of the Declaration of Helsinki and was approved by the Medical Ethics Committee of Chang Gung Memorial Hospital. Because this study was a retrospective review of existing data, Institutional Review Board approval was obtained, but without specific informed consent from the patients. The Institutional Review Board of Chang Gung Memorial Hospital specifically waived the need for consent. The Institutional Review Board number assigned to the study was 202000663B0.
